RETRACTED

# Development of a Relative Similarity Degree Based Engineering Construction Multi-Attribute Decision Model and Its Application

**DOI:** 10.1155/2022/4274795

**Published:** 2022-06-17

**Authors:** Ling Sui, Xiaojie Liang, Qilong Huang

**Affiliations:** No. 501, The Transportation Development Research Center of China Academy of Transportation Sciences, Ministry of Transport R. China, 240 Huixinli, Chaoyang District, Beijing 100029, China

## Abstract

Generally, there are large amounts of uncertain factors in the multi-attribute decision system. By using the gray relational degree and fuzzy gray relational degree, the weights of the comprehensive indexes are extracted. Then, a novel decision model is established based on the concept of relative similarity degree. Finally, comparative research is carried out taking the maritime safety engineering construction in Hunan Province, China, as an example to verify that the developed model is rather effective and practical for its high resolution and sensitivity in multi-attribute decision.

## 1. Introduction

Multi-attribute decision problems refer to selection of the ideal scheme from a limited number of alternative schemes after comprehensively comparing these attributes (indexes) and ranking them in the scheme set. Each attribute in a decision system generally has uncertainty to some extent. Aiming at the presence of these large amounts of uncertain factors, numerous researchers have conducted relevant research. The commonly used method is to extract the weights of indexes to serve the final decision by using the gray relational degree and fuzzy processing method [1, 2]. Literature [3–5] proposed a decision-making method based on possibility and satisfaction, which was improved in literature [6]. Literature [7, 8] gives an integrated method of multiobjective decision-making and extends this method. On this basis, literature [9–15] gives a multi-attribute decision-making method based on distance similarity measure. Literature [16–20] introduces the concept of uncertain fuzzy set and gives an improved method of multiobjective decision-making. Literature [21–23] proposed a new similarity weighted aggregation method.

While these methods can solve practical problems, the obtained decision results show low discreteness and tend to be normalized sometimes, which influences the resolution of the results and the utilization of given information in the system. The above problem becomes more prominent in the comparison of schemes with similar levels, high fuzzy degree, and difficulty in selection. To solve the problem, the concept of relative similarity degree is introduced to construct a novel decision model, followed by comparative research based on a practical case. The research provides a reasonable and effective approach for the comprehensive evaluation of a project.

RETRACTED

## 2. Problem Description

In decision-making problems, in order to ensure the accuracy and effectiveness of decision-making results, the similarity between language terms is a factor that cannot be ignored. In order to better express decision information, the following symbolic notation is used to represent the sets and quantities related to multi-attribute decision-making problems:

 
**X** = {*x*_1_, *x*_2_,…, *x*_*m*_} represents the set of *m* decision schemes
 
**S** = {*s*_1_, *s*_2_,…, *s*_*n*_} refers to the set of *n* attributes which are assumed to be independent
 
**A** = [*a*_*ij*_]_*m × n*_ represents the decision matrix, where *a*_*ij*_ is a result of an attribute *s*_*j*_ using a scheme *x*_*i*_ (i.e., the attribute value)

In general, attributes can be divided into benefit, cost, fixed, and interval types and different attributes possibly have different dimensions. Therefore, for the sake of convenient analysis and calculation, the decision matrix ***A*** needs to be normalized, using the normalization formula in Reference [1] for instance. Suppose that the normalized decision matrix is **B** = [*b*_*ij*_]_*m* *×* *n*_ and $\overset{-}{b_{i}}=\left(1/n\right)\cdot \sum_{j=1}^{n}b_{i,j}$ (*i* = 1,…,*m*) is the expected value of the index.

Let ***ω***_**k**_ = (*ω*_1_, *ω*_2_,…,*ω*_*n*_)^*T*^, where *ω*_*j*_ ≥ 0 (*j* = 1, 2,…, *n*), and ∑_*j*=1_^*n*^*ω*_*j*_=1 is the weight vector of an attribute and *k* denotes the different methods used for extracting the weight. The concepts of ideal point of multiobjective decision-making problem, negative ideal point of multiobjective decision-making problem, and objective vector corresponding to any feasible solution are introduced. It is extracted by gray correlation degree and fuzzy gray correlation degree operator, *k* = 1, 2.

## 3. Establishment of the Multiattribute Decision Model

### 3.1. Extracting Weight *ω*_*j*_ of the Index

Reasonably and correctly extracting the weight of an index is of great significance for investment decision. Theoretically speaking, the larger the influence of an index on other indexes is, the greater the information contained by the index in the system; otherwise, the index has less information. Based on this, the weight of the index is extracted by using the relational operator.

#### 3.1.1. Operator of Gray Relation

In accordance with the gray relational theory, the weight of the *j*th index is defined as follows:

(1) $$\begin{array}{c} \omega_{j}=\frac{\sum_{i=1}^{m}r_{i,j}}{\sum_{j=1}^{n}\sum_{i=1}^{m}r_{i,j}}, \end{array}$$

where

(2) $$\begin{array}{c} r_{i,j}=\frac{\min_{i=1}^{m}\left|b_{i,j}-{\bar{b}}_{i}\right|+\zeta \max_{i=1}^{m}\left|b_{i,j}-{\bar{b}}_{i}\right|}{\left|b_{i,j}-{\bar{b}}_{i}\right|+\zeta \max_{i=1}^{m}\left|b_{i,j}-{\bar{b}}_{i}\right|}\;\left(i=1,\&,m;j=1,\&,n\right), \end{array}$$

is the average gray relational degree. The constant ***ζ*** is the identification coefficient of gray relation. It is used to adjust the size of the comparative environment and generally let it be ***ζ*** = 0.5 in practical engineering applications.

RETRACTED

#### 3.1.2. Operator of Fuzzy Gray Relation

According to the theory of fuzzy system, the weight of the *j*th index is defined as follows:

(3) $$\begin{array}{c} \omega_{j}=\frac{\sum_{i=1}^{m}{\tilde{r}}_{i,j}}{\sum_{j=1}^{n}\sum_{i=1}^{m}{\tilde{r}}_{i,j}}, \end{array}$$

where

(4) $$\begin{array}{c} {\tilde{r}}_{i,j}=\frac{\sum_{i=1}^{m}b_{i,j}\wedge {\bar{b}}_{i}}{\begin{array}{c} \sum_{i}^{m}b_{i,j}\vee {\bar{b}}_{i} \end{array}}. \end{array}$$

### 3.2. Determining the Relative Similarity Degree

Because the relative closeness makes effective use of the distance information from the structural type scheme to the ideal scheme and the negative ideal scheme, the relative closeness method for multi-attribute decision-making can overcome the limitations brought by only using the Euclidean distance. Using the relative closeness between the objective scheme and the ideal point and the satisfaction of the objective function, an interactive multiobjective decision-making method based on relative closeness is proposed as follows:

(1) Constructing the expanded normalized decision matrix *C*
Optimal and worst schemes are the possible ideal and least ideal schemes in a comprehensive evaluation problem.
Assume that the optimal and worst schemes are $\bar{P}$ = {*p*_1_, *p*_2_,…, *p*_*n*_} (*p*_*j*_ ≥ 0) and $\bar{Q}$ = { *q*_1_, *q*_2_,…, *q*_*n*_} (*q*_*j*_ ≥ 0), respectively.
After normalization of the index, the normalized decision matrix **B** = [*b*_*ij*_]_*m* *×* *n*_ is obtained, in which 0 ≤ *b*_*ij*_ ≤ 1 and the larger the value of *b*_*ij*_ is, the better a scheme under the current index. Obviously, the optimal scheme in the decision matrix **B** is when the values of all of the normalized indexes are 1, and the worst scheme is when the values of the normalized indexes are 0. While as a matter of fact, these two schemes are difficult to obtain. However, to extract the relative similarity degree, the optimal and worst schemes are also considered, that is, adding two rows (all indexes valuing 1 and 0, separately) in the matrix **B**, thus obtaining the following expanded normalized decision matrix *C*:
  (5) $$\begin{array}{c} C=\left[\begin{array}{cccc} c_{11} & c_{12} & \cdots & c_{1n}\\ c_{21} & c_{22} & \cdots & c_{2n}\\ \cdots & \cdots & \cdots & \cdots \\ c_{m1} & c_{m2} & \cdots & c_{mn}\\ 1 & 1 & \cdots & 1\\ 0 & 0 & \cdots & 0 \end{array}\right]. \end{array}$$
(2) Weights are assigned to the expanded normalized decision matrix *C*, to attain the following weighted expanded normalized matrix *D*:
  (6) $$\begin{array}{c} D=\begin{array}{c} x_{1}\\ x_{2}\\ \cdots \\ x_{m}\\ \bar{P}\\ \bar{Q} \end{array}\left[\begin{array}{cccc} d_{11} & d_{12} & \cdots & d_{1n}\\ d_{21} & d_{22} & \cdots & d_{2n}\\ \cdots & \cdots & \cdots & \cdots \\ d_{m1} & d_{m2} & \cdots & d_{mn}\\ \omega_{1} & \omega_{2} & \cdots & \omega_{n}\\ 0 & 0 & \cdots & 0 \end{array}\right]\\ =\left[\begin{array}{cccc} \omega_{1}c_{11} & \omega_{2}c_{12} & \cdots & \omega_{n}c_{1n}\\ \omega_{1}c_{21} & \omega_{2}c_{22} & \cdots & \omega_{n}c_{2n}\\ \cdots & \cdots & \cdots & \cdots \\ \omega_{1}c_{m1} & \omega_{2}c_{m2} & \cdots & \omega_{n}c_{mn}\\ \omega_{1} & \omega_{2} & \cdots & \omega_{n}\\ 0 & 0 & \cdots & 0 \end{array}\right]. \end{array}$$
(3) Determining the ideal point *E*^+^ and the negative ideal point *E*^−^
  (7) $$\begin{array}{c} E^{+}=\max_{i}\left\{d_{ij}|j=1,2,\ldots ,n\right\}\\ =\left(E_{1}^{+},E_{2}^{+},\ldots ,E_{n}^{+}\right),\\ E^{-}=\max_{j}\left\{d_{ij}|j=1,2,\ldots ,n\right\}\\ =\left(E_{1}^{-},E_{2}^{-},\ldots ,E_{n}^{-}\right). \end{array}$$
It can be seen from the matrix *D* that *E*^*+*^ = (*ω*_1_, *ω*_2_,…, *ω*_*n*_) and *E*^−^ = (0, 0,…, 0).
(4) Calculating the relative similarity degree of each scheme with the ideal point:
  (8) $$\begin{array}{c} \frac{\left(E^{+}-D_{i}\right){\left(E^{+}-E^{-}\right)}^{T}}{{\left\|E^{+}-E^{-}\right\|}^{2}}=1-\frac{\sum_{j}^{n}\omega_{j}d_{ij}}{\sum_{j}^{n}\omega_{j}^{2}},\;i=1,2,\ldots ,m, \end{array}$$

where *D*_*i*_ = (*d*_*i*1_, *d*_*i*2_,…, *d*_*in*_).

RETRACTED

The value of *T*_*i*_ reflects the similarity degree of a scheme with the ideal scheme and the disparity with the worst scheme, that is, the relative similarity degree with the ideal point. Apparently, *T* ∈ [0, 1]. The smaller the value of *T*_*i*_ is, the more similar a decision scheme with the ideal point and, correspondingly, the better the scheme; otherwise, the scheme is worst.

### 3.3. Establishing the Decision Model

In general conditions, the decision model for multi-attribute problems based on gray relation and fuzzy gray relation is as follows:

(9) $$\begin{array}{c} Y_{i}=\sum_{j}^{n}\omega_{j}\circ b_{ij},\;i=1,2,\ldots ,m, \end{array}$$

where ○ represents a certain operation and *Y*_*i*_ is the array output from the decision results. The larger the value of *Y*_*i*_ is, the better the scheme.

According to the above analysis, the relative similarity degree based decision model is constructed as follows:

(10) $$\begin{array}{c} Y_{i}=1-\frac{\sum_{j}^{n}\omega_{j}d_{ij}}{\sum_{j}^{n}\omega_{j}^{2}},\;i=1,2,\ldots ,m, \end{array}$$

where *Y*_*i*_ represents the output array of the decision results. The scheme with a smaller value of *Y*_*i*_ is more similar to the ideal point; that is, the scheme is better.

## 4. Case Study

To verify the model established in the research, several decision models for the construction and planning of maritime safety engineering in Hunan Province, China, were compared based on the self-designed investment decision support system of maritime safety engineering construction. Taking the construction planning of Maritime Safety Engineering in Hunan Province as an example, the decision-making models of gray correlation degree, fuzzy gray correlation degree, and relative closeness degree are used for comparative research.

From the perspective of the optimal comprehensive benefit of the construction project of local maritime safety engineering, the index system (the RAW data were derived from the *Construction and Planning Report for the Maritime Safety Engineering in Cities of Hunan Province, China* (November, 1999)) for comprehensive evaluation is constructed (Table 1). The 17 technical and economic indexes (attributes) in the table involve multiple aspects including the technology, economy, environment, and society. By conducting a preliminary feasibility study and expert survey, most of these attributes are benefit-type except for the investment volume per unit length of river bank and the buildings demolished for building per unit length of river bank which are cost-type attributes.

At first, the range transformation method is used to normalize the indexes. Then, the weights ***ω***_**1**_ and ***ω***_**2**_ of the index based on gray relational degree and fuzzy gray relational degree are obtained by using (1) and (3), respectively [4].

 
***ω***_**1**_ = (0.0593 0.0523 0.0583 0.0649 0.0626 0.0611 0.0701 0.0685 0.0615 0.0555 0.0525 0.0474 0.0594 0.0576 0.0556 0.0583 0.055)^*T*^
 
***ω***_**2**_ = (0.0531 0.0342 0.0514 0.0794 0.0618 0.0694 0.0862 0.0805 0.0744 0.0579 0.0614 0.0175 0.0546 0.0569 0.0423 0.063 0.056)^*T*^

The decision results in Table 2 are obtained by using (9).

The decision results in Table 3 are acquired by using (10).

It can be seen from the above case study that the results obtained using different decision models are basically consistent; that is, Changsha applies the optimal scheme while Zhangjiajie uses the worst one. Using the decision-making methods of gray correlation degree and fuzzy gray correlation degree, a decision-making model of correlation degree is constructed based on the concepts of interval gray and fuzzy gray, but the correlation degree with the ideal scheme is not considered, so the scheme ranking may be one-sided. The decision-making method of relative closeness degree integrates the relevance closeness degree and can comprehensively consider the relationship between each scheme and positive and negative ideal schemes, so that the decision-making will not deviate from the phenomenon and is more practical. It is not difficult to find from the analysis results and the decision results (Table 2) obtained using the method based on the relative similarity degree are more discrete and have more sensitive ranking, so it is more beneficial to the decision of the scheme, in comparison with the results (Table 3) attained using the other method. It indicates that the decision model based on the relative similarity degree is particularly suitable for situations with schemes of little discrepancies and requiring more elaborate and reliable decision.

RETRACTED

## 5. Conclusions

Based on the developed investment decision support system of maritime safety engineering construction, the multi-attribute decision model based on the concept of relative similarity degree is used to carry out numerous case studies. The decision results obtained are objective, which verifies the effectiveness and rationality of the model. Compared with the existing gray relational decision-making model, this decision-making method can comprehensively consider the relationship between each scheme and positive and negative ideal schemes, so that the decision-making will not deviate. With clear concept and reasonable logic and making full use of the decision information of the system, the proposed model is capable of improving the sensitivity and resolution of the decision results and, therefore, is an effective method for solving multi-attribute decision problems. It is worth noting that apart from the two methods for extracting weights of indexes proposed in the research, other methods can also be used to extract weight. By combining with the relative similarity degree, these methods can also meet the requirement for improving the identification precision. Considering the difficulty of sharing multiple attributes of indicators in decision-making and the multidimensional fit between the alternative and the ideal scheme, further optimize and improve the model to improve the identification and sensitivity of decision-making.

## Figures and Tables

**Table 1:** Technical and economic indexes for the construction and planning of maritime safety engineering in cities of Hunan province.

City	Internal rate of return (%)	Net present value (1 × 10^8^ yuan)	Benefit-cost ratio	Affected population (10,000 people)	Area of flooded cultivated land (10,000 hectares)	Direct economic loss (1 × 108 yuan)	Urban Population (10,000 people)	Urban construction area (km^2^)	Gross fixed assets (1 × 108 yuan)

Changsha	16.2	6.5018	1.47	51.2	0.82	83.84	132.43	115	303.6
Changde	18	5.9223	1.63	55.45	1.65	106	55.45	35.3	144
Zhangjiajie	14.43	0.4894	1.26	3.888	0.0000625	0.2079	12.96	12.5	26
Yiyang	13.4	0.46	1.14	22.4	0.032	13.4	45.9	29.5	106
Yueyang	14.0	1.073	1.21	22	0.3887	18.544	65.17	55	162.8
Zhuzhou	15.3	1.1818	1.34	24.522	0.1841	87.84	71.19	58	277.3
Hengyang	14.5	1.2183	1.26	19.5	0.4373	18.6	54.17	46	234
Xiangtan	23.6	7.1305	2.31	32.6	0.526	50.4	65	40	122

City	GDP per capita (yuan)	Growth factor of maritime safety criterion	Growth factor of conservation criterion	Population in the planning area protected by unit project quantity (10,000 people)	Planning area protected by unit project quantity (km^2^)	Investment volume for unit project quantity (10,000 yuan)	Buildings demolished for building unit project quantity (10,000 m^2^)	Environmental benefit coefficient	

Changsha	39354.84	10.43	0.4286	0.6217	0.5238	651.4353	0.2071	9	
Changde	13201.08	10.76	0.3333	0.5454	1.7935	889.7941	0.2293	9	
Zhangjiajie	36010.80	9	9	0.6906	0.8978	659.9275	0.2869	5	
Yiyang	18540.31	10.11	0.6667	1.4061	2.4332	779.9513	0.1572	5	
Yueyang	31497.24	2.33	0.3333	3.8601	4.1780	1463.3565	0.1558	8	
Zhuzhou	27081.05	4.71	0.5385	1.7704	1.7499	840.8024	0.2734	6	
Hengyang	15320.69	4.71	0.8182	1.0196	0.8413	683.3180	0.0985	7	
Xiangtan	14300	4.71	1.5	0.9942	0.9942	671.2281	0.1146	7	

RETRACTED

**Table 2:** Decision results obtained using the two different methods.

	Changsha (%)	Changde (%)	Zhangjiajie (%)	Yiyang (%)	Yueyang (%)	Zhuzhou (%)	Hengyang (%)	Xiangtan (%)
***ω***_**1**_	61.56	49.15	21.70	21.47	41.96	39.80	22.30	39.80
***ω***_**2**_	67.03	53.03	19.90	23.63	42.70	43.37	24.46	39.17

**Table 3:** Decision results based on the relative similarity degree.

	Changsha (%)	Changde (%)	Zhangjiajie (%)	Yiyang (%)	Yueyang (%)	Zhuzhou (%)	Hengyang (%)	Xiangtan (%)
***ω***_**1**_	37.03	50.24	80.18	78.54	57.78	59.29	77.01	60.04
***ω***_**2**_	27.65	44.79	82.34	75.11	57.60	53.64	73.27	61.36

## Data Availability

The original data come from the construction planning report of urban maritime safety projects in Hunan Province in November 1999. Some data, such as the total urban population, urban construction area, and total value of fixed assets, come from the Statistical Yearbook of National Economic and Social Development of Hunan Province in that year. The data are all paper and are not published on the Internet, so they cannot be linked. However, the data and research results of this paper can be cited publicly.
